# Fuzzy PID Control for Respiratory Systems

**DOI:** 10.1155/2021/7118711

**Published:** 2021-06-24

**Authors:** Ibrahim M. Mehedi, Heidir S. M. Shah, Ubaid M. Al-Saggaf, Rachid Mansouri, Maamar Bettayeb

**Affiliations:** ^1^Department of Electrical and Computer Engineering (ECE), King Abdulaziz University, Jeddah 21589, Saudi Arabia; ^2^Center of Excellence in Intelligent Engineering Systems (CEIES), King Abdulaziz University, Jeddah 21589, Saudi Arabia; ^3^Laboratoire de Conception et Conduite des Systemes de Production (L2CSP), Tizi Ouzou, Algeria; ^4^Electrical Engineering Department, University of Sharjah, Sharjah, UAE

## Abstract

This paper presents the implementation of a fuzzy proportional integral derivative (FPID) control design to track the airway pressure during the mechanical ventilation process. A respiratory system is modeled as a combination of a blower-hose-patient system and a single compartmental lung system with nonlinear lung compliance. For comparison purposes, the classical PID controller is also designed and simulated on the same system. According to the proposed control strategy, the ventilator will provide airway flow that maintains the peak pressure below critical levels when there are unknown parameters of the patient's hose leak and patient breathing effort. Results show that FPID is a better controller in the sense of quicker response, lower overshoot, and smaller tracking error. This provides valuable insight for the application of the proposed controller.

## 1. Introduction

The world has been shocked by the COVID-19 disease since its outbreak was first detected in Wuhan, China, in December 2019. It was then declared as a global pandemic by the World Health Organization (WHO) three months later, and at the time of writing, more than 174 million people worldwide have been infected with the disease with close to 4 million deaths recorded [1, 2]. The analysis shows that acute respiratory failure (ARF) is the leading cause of death [3], and one study found that 40 percent of critically ill COVID-19 patients developed acute respiratory distress syndrome (ARDS) which requires invasive incubation and ventilation [4–7]. Such therapies can be provided by an intensive care unit's (ICU) device called a mechanical ventilator that is used to assist or replace the spontaneous breathing of a patient [8].

Mechanical ventilators were first used to assist in ventilation as early as the 18th century, but the first closed-loop system for mechanical ventilation did not become available until the 1950s. A mechanical ventilator used mechanical bellows and valves to cycle gas into the lungs, while a simple proportional (P) or proportional-integral (PI) controller was used [9]. Later, microprocessors were used to implement those controllers, and since then, there have been numerous closed-loop control proposals.

Closed-loop control in mechanical ventilators can be categorized based on how much the system interacts with patients. A class 1 control loop features no backward interaction from the patient to the device, whereas in the class 2 control loop, interaction between the patient and device is possible. In both classes, control signals are measured inside the device. A class 3 control loop is called *physiological compensatory control loops* due to the fact that it uses the physiological parameter as its control variable instead of the physical one [10]. In this paper, a pressure-based ventilation controller under the class 2 category is developed where the control objective is to track a set-point target airway pressure.

Having a reputation as the most reliable industrial controller, the PID controller has been used widely in mechanical ventilators. One of the earliest implementations of PID controller on a mechanical ventilator since the introduction of the microprocessor can be found in *Ohlson* works [11]. PID, however, has some limitations: it did not perform well when the system's dynamics are not constant. An example of this is the relationship between ventilation and pressure. During ventilation, pressure must be adjusted according to the level of ventilation to prevent lung injury. To improve controller performance, Dai et al. [12] used two separate algorithms where the PD algorithm is used during the initial phase while PI algorithm will be activated when the output pressure started to be constant. Besides this, other techniques were also used to improve PID controller performance in the mechanical ventilation system including the use of optimization techniques called pressure evaluate correction module (PECM) [13], an automatic tuning of PID gains using particle swarm optimization (PSO) [14, 15] and repetitive control [8].

In this paper, we proposed a fuzzy PID (FPID) controller for airway pressure set-point tracking of mechanical ventilation. Fuzzy reasoning is used to evaluate the changes of the system's dynamic through the measured set-point error and the rate of change of error which, in turn, updates the PID tuning parameters based on the rules set. The process of updating the tuning parameters is done in an online manner. The proposed controller is then simulated on a respiratory system model which consists of a blower-hose-patient system model and a single compartmental lung model which is obtained from the works of Hunnekens et al. [16] and Bates [17], respectively.

The fuzzy logic-based controller has been implemented in many applications including the longitudinal autopilot of an unmanned aerial vehicle (UAV) [18], controlling the speed of the conveyor system [19], simulating the tissue differentiation process [20], and induction motor control [21]. The primary purpose of this proposed controller is to enhance the performance of the PID controller on a respiratory system where some of its mechanical parameters are not constant, specifically, lung compliance, which can be increased or decreased according to the lung volume.

The rest of this paper is organized as follows: Section 2 presents the details of the mathematical model for the blower-hose-patient system and single lung compartmental model and also presents a brief explanation about lung compliance. The details of the proposed controller design are discussed in Section 3, while the simulation results, analysis, and comparison between PID and FPID are presented in Section 4.  Section 5 concludes the work.

## 2. Mathematical Model of Respiratory Systems

The respiratory system model used in this paper is based on the blower-hose-patient system model presented in [16] with a single compartmental lung model obtained from [17]. As shown in Figure 1, the system consists of 3 main components: the blower which compresses ambient air to the desired pressure, (*p*_out_), the hose which connects the respiratory module to the patient, and the patient's lung. The airway pressure *p*_*aw*_ is measured using a pressure sensor that is placed inside the module. The control objective is to track the measured pressure so that it follows the target set-point *p*_target_. Therefore, the error equation can be described as follows:

(1) $$\begin{array}{c} e=p_{\text{target}}-p_{\text{aw}}. \end{array}$$

The air from the blower flows (*Q*_out_) through the hose with the resistance of *R*_hose_ into the lung (*Q*_pat_) with the resistance of *R*_lung_ for inhalation process. The patient then exhales the air back to the hose where some of it will flow out of the leak (*Q*_leak_) with the resistance of *R*_leak_. The leak also prevents some of the exhaled air to be inhaled back by the patient in the next cycle. Thus, we can write the patient flow equation as follows:

(2) $$\begin{array}{c} Q_{\text{pat}}=Q_{\text{out}}-Q_{\text{leak}}, \end{array}$$

Here, the blower flow, leak flow, and patient flow can be obtained by pressure differences over resistance as follows:

(3) $$\begin{array}{c} Q_{\text{out}}=\frac{p_{\text{out}}-p_{aw}}{R_{\text{hose}}}, \end{array}$$

(4) $$\begin{array}{c} Q_{\text{leak}}=\frac{p_{aw}}{R_{\text{leak}}}, \end{array}$$

(5) $$\begin{array}{c} Q_{\text{pat}}=\frac{p_{aw}-p_{\text{lung}}}{R_{\text{lung}}}. \end{array}$$

The lung pressure can be described by the following differential equation:

(6) $$\begin{array}{c} {\dot{p}}_{\text{lung}}=\frac{1}{C_{\text{lung}}}Q_{\text{pat}}. \end{array}$$

The lung dynamic can be written by combining (3)–(6) as follows:

(7) $$\begin{array}{c} {\dot{p}}_{\text{lung}}=\frac{p_{aw}-p_{\text{lung}}}{C_{\text{lung}}R_{\text{lung}}}. \end{array}$$

Substituting and rewriting (3)–(5) in (2) results in the following relation for the airway pressure:

(8) $$\begin{array}{c} p_{aw}=\frac{\left(1/R_{\text{lung}}\right)p_{\text{lung}}+\left(1/R_{\text{hose}}p_{\text{out}}\right)}{\left(1/R_{\text{lung}}\right)+\left(1/R_{\text{hose}}\right)+\left(1/R_{\text{leak}}\right)}. \end{array}$$

By substituting the airway pressure expression in (8) into the differential equation for the lung dynamic (6), the following may be achieved:

(9) $$\begin{array}{c} {\dot{p}}_{\text{lung}}=\frac{-\left(\left(1/R_{\text{hose}}\right)+1/R_{\text{leak}}\right)p_{\text{lung}}+\left(1/R_{\text{hose}}\right)p_{\text{out}}}{R_{\text{lung}}C_{\text{lung}}\left(\left(1/R_{\text{lung}}\right)+\left(1/R_{\text{hose}}\right)+\left(1/R_{\text{leak}}\right)\right)}. \end{array}$$

Now, equations (5), (7), and (8) can be arranged into a state-space form with *p*_out_ as input, [*p*_aw_, *Q*_pat_]^*T*^ as outputs, and *p*_lung_ as state:

(10) $$\begin{array}{c} {\dot{p}}_{\text{lung}}=A_{h}p_{\text{lung}}+B_{h}p_{\text{out}}, \end{array}$$

(11) $$\begin{array}{c} \left[\frac{p_{aw}}{Q_{\text{pat}}}\right]=C_{h}p_{\text{lung}}+D_{h}p_{\text{out}}, \end{array}$$

where

(12) $$\begin{array}{c} A_{h}=-\frac{\left(1/R_{\text{hose}}\right)+\left(1/R_{\text{leak}}\right)}{R_{\text{lung}}C_{\text{lung}}\left(\left(1/R_{\text{lung}}\right)+\left(1/R_{\text{hose}}\right)+\left(1/R_{\text{leak}}\right)\right)},\\ B_{h}=\frac{\left(1/R_{\text{hose}}\right)}{R_{\text{lung}}C_{\text{lung}}\left(\left(1/R_{\text{lung}}\right)+\left(1/R_{\text{hose}}\right)+\left(1/R_{\text{leak}}\right)\right)},\\ C_{h}={\left[\begin{array}{cc} \frac{\left(1/R_{\text{lung}}\right)}{\left(1/R_{\text{lung}}\right)+\left(1/R_{\text{hose}}\right)+\left(1/R_{\text{leak}}\right)} & -\frac{\left(1/R_{\text{hose}}\right)+\left(1/R_{\text{leak}}\right)}{R_{\text{lung}}\left(\left(1/R_{\text{lung}}\right)+\left(1/R_{\text{hose}}\right)+\left(1/R_{\text{leak}}\right)\right)} \end{array}\right]}^{T},\\ D_{h}={\left[\begin{array}{cc} \frac{\left(1/R_{\text{hose}}\right)}{\left(1/R_{\text{lung}}\right)+\left(1/R_{\text{hose}}\right)+\left(1/R_{\text{leak}}\right)} & \frac{\left(1/R_{\text{hose}}\right)}{R_{\text{lung}}\left(\left(1/R_{\text{lung}}\right)+\left(1/R_{\text{hose}}\right)+\left(1/R_{\text{leak}}\right)\right)} \end{array}\right]}^{T}. \end{array}$$

A state-space model of the blower, however, can be expressed as follows:

(13) $$\begin{array}{c} {\dot{x}}_{b}=A_{b}x_{b}+B_{b}p_{\text{control}}, \end{array}$$

(14) $$\begin{array}{c} p_{\text{out}}=C_{b}x_{b}. \end{array}$$

By coupling expression in (10), (13), and the respiratory system (14), the general state-space model for the respiratory system is obtained:

(15) $$\begin{array}{c} {\dot{x}}_{p}=\left[\frac{{\dot{x}}_{b}}{{\dot{p}}_{\text{lung}}}\right]=\left[\begin{array}{cc} 0 & A_{b}\\ B_{h}C_{b} & A_{h} \end{array}\right]\left[\frac{x_{b}}{p_{\text{lung}}}\right]+\left[\frac{B_{b}}{0}\right]p_{\text{control}}. \end{array}$$

Equation (6) shows that one of the factors that determine the dynamic of the lung pressure is a parameter called lung compliance (*C*_lung_). It is a measure of the change in lung volume per change in transpulmonary pressure, or in simpler words, the ease at which the lung can expand under pressure. Clinical data show that lung compliance values are not constant all the time and sometimes increases or decreases according to the lung volumes. The value can, however, be constant when a certain transition region of lung volume is entered [22].

## 3. Controller Design

The structure of the PID controller is shown in Figure 2, where three parameters—proportional gain *K*_*p*_, integral gain *K*_*i*_, and derivative gain *K*_*d*_—are used to manually tune the controller. The output of the controller is the blower's pressure which is given by the following equation:

(16) $$\begin{array}{c} p_{\text{out}}=K_{p}e\left(t\right)+K_{i}\int_{0}^{t}e\left(t\right)\text{dt}+K_{d}\frac{\text{d}e\left(t\right)}{\text{d}t}, \end{array}$$

where

(17) $$\begin{array}{c} K_{i}=K_{p}\frac{T_{s}}{T_{i}}, \end{array}$$

(18) $$\begin{array}{c} K_{d}=K_{p}\frac{T_{d}}{T_{s}}. \end{array}$$

*T*_*i*_ and *T*_*d*_ in equations (17) and (18) is the integral and derivative time, respectively, while *T*_*s*_ is the sampling time. Ciancone correlation technique with fine tuning is used to tune the PID parameters. The PID parameter's value obtained is *K*_*p*_=1.1 × 10^−3^, *K*_*i*_=12 × 10^−3^, and *K*_*d*_=15 × 10^−6^.

In fuzzy PID controller whose structure is shown in Figure 3, a fuzzy inference system (FIS) is used to tune all the three PID parameters. The input to the FIS is the error *e* and the rate of change of error Δ*e*, while the output is the PID parameters *K*_*p*_, *K*_*i*_, and *K*_*d*_, where their initial values are the same as the ones previously obtained via Ciancone correlation. Each of the inputs and outputs consists of 3 membership functions labeled as negative (N), zero (Z), and positive (P). The range of values for these functions was determined from the experience in manually tuning the PID controller. Figures 4 and 5 show the membership function used for the input and output of the FIS, respectively.

The value of PID parameters was determined based on the following 4 basic rules:

1. When *e* is large and Δ*e* is negative, the system's response is still far from the set-point through its heading towards the right direction. Therefore, *K*_*p*_ must be large, while *K*_*i*_ and *K*_*d*_ should be small to quickly close in with the set-point.
2. When *e* is negative and Δ*e* is large, the system's response has surpassed the set-point and the error is rising. *K*_*d*_ is set to large, while *K*_*i*_ and *K*_*p*_ are set to small in order to limit the overshoot.
3. When *e* is small, and Δ*e* is positive, the system's response is closing in steady-state. Therefore, *K*_*p*_ should be big to reach steady-state quickly; however, to decrease the overshoot and avoid oscillation, *K*_*d*_ should be added while *K*_*i*_ should be diminished.
4. When *e* is large and Δ*e* is positive, the system's response is overshooting at the negative side. *K*_*d*_ should be large to reduce the error, while *K*_*p*_ and *K*_*i*_ should also increase.

The complete fuzzy rules for the system are as shown in Tables 1–3.

## 4. System's Simulations and Results

The performances of the controller developed in Section 3 are evaluated by simulating it on the model described in Section 3. Integral time absolute error (ITAE) shown as follows is used to measure the set-point tracking performance of both controllers.

(19) $$\begin{array}{c} \text{ITAE}=\int_{0}^{x}t\left|e\left(t\right)\right|\text{dt}. \end{array}$$

The maximum target pressure *p*_target_ is set at 20*mbar*, and the following system's parameters were used in the simulation: *R*_Lung_=0.005 mbar/*mL*/*s*, *R*_Leak_=0.06 mbar/*mL*/*s*, and *R*_hose_=0.0045 mbar/*mL*/*s*. First, we simulate the PID controller on two different lung compliance values, one with constant 20  *mL*/mbar throughout the inhalation and exhalation process and the other as a function of lung volume as shown in Figure 6.

The results in Figure 7 show that it is more difficult to track the pressure set-point with the lung compliance value changing with lung volumes. Under this condition, the controller responses with more oscillation and higher overshoot as compared with when the PID controller is simulated in the model with constant lung compliance value.

Fuzzy PID controller is then simulated using the same parameters and the results as compared to the PID controller which is illustrated in Figure 8. Here, we can observe that FPID has a quicker response and lower overshoot. FPID controller is also better at tracking the set-point based on the calculated ITAE where FPID scored 7.467 while PID scored 8.293.

## 5. Conclusion

This paper has presented the simulation results of applying FPID control design in a pressure-based mechanical ventilation system. The respiratory system was modeled by combining the blower-hose-patient system with a single compartmental lung system with nonlinear lung compliance. It has been shown in the simulation results that the poor performance of the PID controller in tracking the airway pressure of the modeled system can be improved by applying fuzzy reasoning to tune the PID parameters online automatically. The performance was improved in terms of quicker response, lower overshoot, and small tracking error (ITAE). However, there is still some room for improvement. Further study on the number and type of membership function used in the FIS could improve the performance further.

## Figures and Tables

**Figure 1:** Blower-hose-patient system.

**Figure 2:** PID control of the respiratory system.

**Figure 3:** Fuzzy PID control of the respiratory system.

**Figure 4:** Membership function for error *e* and Δ*e*.

**Figure 5:** Membership function for *K*_*p*_, *K*_*i*_, and *K*_*d*_.

**Figure 6:** Compliance function.

**Figure 7:** PID controller response on respiratory system with constant vs. nonlinear compliance value.

**Figure 8:** PID vs. FPID controller response.

**Table 1:** Fuzzy rules for *K*_*p*_.

*K*_*p*_		Δ*e*		
		**N**	**Z**	**P**
**e**	**N**	*N*	*Z*	*N*
	**Z**	*Z*	*Z*	*Z*
	**P**	*P*	*Z*	*P*

**Table 2:** Fuzzy rules for *K*_*i*_.

*K*_*i*_		Δ*e*		
		**N**	**Z**	**P**
**e**	**N**	*N*	*Z*	*N*
	**Z**	*Z*	*Z*	*N*
	**P**	*N*	*Z*	*P*

**Table 3:** Fuzzy rules for *K*_*d*_.

*K*_*d*_		Δ*e*		
		**N**	**Z**	**P**
**e**	**N**	*N*	*Z*	*N*
	**Z**	*Z*	*Z*	*N*
	**P**	*N*	*Z*	*P*

## Data Availability

No data were used to support this study.
